This article has been retracted.

# Characteristics of liver fibrosis with different etiologies using a fully quantitative fibrosis assessment tool

**DOI:** 10.1590/1414-431X20175234

**Published:** 2017-05-18

**Authors:** Q. Wu, X. Zhao, H. You

**Affiliations:** 1 Beijing Key Laboratory of Translational Medicine in Liver Cirrhosis, Liver Research Center, Beijing Friendship Hospital, Capital Medical University, Beijing, China; 2 National Clinical Research Center for Digestive Diseases, Beijing, China

**Keywords:** Liver fibrosis, Quantitative assessment, Etiology

## Abstract

This study aimed to test the diagnostic performance of a fully quantitative fibrosis assessment tool for liver fibrosis in patients with chronic hepatitis B (CHB), primary biliary cirrhosis (PBC) and non-alcoholic steatohepatitis (NASH). A total of 117 patients with liver fibrosis were included in this study, including 50 patients with CHB, 49 patients with PBC and 18 patients with NASH. All patients underwent liver biopsy (LB). Fibrosis stages were assessed by two experienced pathologists. Histopathological images of LB slices were processed by second harmonic generation (SHG)/two-photon excited fluorescence (TPEF) microscopy without staining, a system called qFibrosis (quantitative fibrosis) system. Altogether 101 quantitative features of the SHG/TPEF images were acquired. The parameters of aggregated collagen in portal, septal and fibrillar areas increased significantly with stages of liver fibrosis in PBC and CHB (P<0.05), but the same was not found for parameters of distributed collagen (P>0.05). There was a significant correlation between parameters of aggregated collagen in portal, septal and fibrillar areas and stages of liver fibrosis from CHB and PBC (P<0.05), but no correlation was found between the distributed collagen parameters and the stages of liver fibrosis from those patients (P>0.05). There was no significant correlation between NASH parameters and stages of fibrosis (P>0.05). For CHB and PBC patients, the highest correlation was between septal parameters and fibrosis stages, the second highest was between portal parameters and fibrosis stages and the lowest correlation was between fibrillar parameters and fibrosis stages. The correlation between the septal parameters of the PBC and stages is significantly higher than the parameters of the other two areas (P<0.05). The qFibrosis candidate parameters based on CHB were also applicable for quantitative analysis of liver fibrosis in PBC patients. Different parameters should be selected for liver fibrosis assessment in different stages of PBC compared with CHB.

## Introduction

The severity of liver fibrosis is an important factor for long-term prognosis of liver disease. Studies show that liver fibrosis is a reversible process (1 [Bibr B02]–3). Accurate and quantitative assessment of liver fibrosis is very important in diagnosis, treatment and prognosis of liver disease.

Liver biopsy is still the gold standard for quantitative assessment of liver fibrosis. From the initial subjective and descriptive diagnosis to the current semi-quantitative score system, the pathological assessment of liver fibrosis has improved greatly. Several semi-quantitative staging systems exist, including Knodell staging system, Ishak staging system, Metavir staging system, and others (4). Although semi-quantitative diagnosis is more convenient for clinical practitioners compared with the initial descriptive diagnosis, those methods are still not very reliable and repeatable because the results depend on the staining process.

Noninvasive diagnostic methods for liver fibrosis, including fibroscan and MRI, have been widely used in the diagnosis of severe liver fibrosis and cirrhosis in recent years, but these methods are not effective in the diagnosis of mild or moderate liver fibrosis. So currently, the noninvasive diagnostic methods can not completely substitute liver biopsy (5).

In recent years, a new concept of quantitative structure has been proposed, which is based on a new technology tool – qFibrosis analysis system (6). It relies on non-linear second harmonic generation (SHG)/two-photon excitation fluorescence (TPEF) microscopy imaging technique. Combining organizational engineering, biophotonics and clinical liver disease theory and technology, qFibrosis can faithfully replicate traditional fibrosis score and detect subtle quantitative fibrosis changes (7 [Bibr B08] [Bibr B09]–10 [Bibr B11]). SHG/TPEF can analyze and quantify collagen fibers because it is very sensitive in detecting dissymmetry in the structure of fibrillar collagen molecules in stain-free biopsy sections. This quantitative method for liver fibrosis evaluation is supposedly superior than traditional semi-quantitative staging systems for it is objective, fully quantitative, less sensitive to sampling error, and can mediate inter-/intra-observer variation (6). The method has been recently validated in chronic hepatitis B (6). However, its accuracy to detect extensive fibrosis or cirrhosis in other chronic liver diseases remains to be demonstrated.

The aim of this study is to assess the diagnostic performance of qFibrosis for the evaluation of fibrosis and histological stages in chronic cholestatic diseases of primary biliary cirrhosis (PBC) and non-alcoholic steatohepatitis (NASH) by comparing with the results from chronic hepatitis B (CHB), to analyze the characteristics of different etiology liver fibrosis in different stages, and to provide theoretical basis and data for further clinical application of qFibrosis.

## Material and Methods

### Patients

Altogether 117 patients with liver fibrosis, including 50 patients with chronic hepatitis B (CHB), 49 patients with primary biliary cirrhosis (PBC), and 18 patients with non-alcoholic steatohepatitis (NASH) were retrospectively enrolled from October 2010 to October 2015, in Beijing Friendship Hospital, Capital Medical University. Patients diagnosed with a single known etiology and that underwent percutaneous liver biopsy (LB) were included in this study. Patients with other or mixed etiologies, and malignancy were excluded. Informed written consent was obtained from all patients and the study was approved by the Research Ethics Committee of the Beijing Friendship Hospital.

PBC was defined according to the 2009 PBC practice guidelines from the American Association for the Study of Liver Diseases (AASLD) (12), as follows: biochemical evidence of cholestasis based mainly on alkaline phosphatase elevation; presence of antimitochondrial antibodies; histological evidence of nonsuppurative destructive cholangitis and destruction of interlobular bile ducts. NASH was defined according to the 2012 Practice Guideline by the American Astroenterological Association (AGA), AASLD, and American College of Gastroenterology (ACG): The Diagnosis and Management of Non-alcoholic Fatty Liver Disease Practice Guideline (13).

### Liver histology

Liver biopsy specimens were routinely fixed in formalin and paraffin embedded. Five-micron thick sections were stained with Masson trichrome for histological assessment. Biopsy specimens were analyzed independently by two experienced pathologists. Liver fibrosis of CHB and PBC were evaluated semiquantitatively according to the Metavir staging system (14): F0: no fibrosis; F1: stellate enlargement of portal tracts but without septum formation; F2: enlargement of portal tracts with rare septum formation; F3: numerous septa without cirrhosis; F4: cirrhosis. NASH fibrosis was classified into 5 stages: stage 0: no fibrosis; stage 1: mild or moderate zone 3 perisinusoidal fibrosis; stage 2: perisinusoidal fibrosis enlarged to portal stellate fibrosis; stage 3: bridging fibrosis; stage 4: cirrhosis.

### SHG/TPEF microscopy imaging and processing

The embedded biopsy specimen sectioned at 5-μm thickness were dewaxed for imaging by the SHG/TPEF microscopy system (HistoIndex, Genesis 200¯, Singapore). Collagen was visualized by SHG microscopy and hepatocyte morphology was acquired by the TPEF microscopy. We used the full scan method to acquire the images. Images were acquired at 20× magnification with 512×512 pixel resolutions. Image processing and analysis (threshold and SHG scoring) were routinely performed, and 101 quantitative morphological features of the SHG/TPEF image were acquired by the computer-aided system. Three main fibrosis patterns – collagen in portal area (portal expansion), collagen in septal area (bridging fibrosis), and collagen in fibrillar area (fine collagen distributed in the pericellular/perisinusoidal space – or space of Disse) were evaluated in this study. Collagen features were classified into three groups: collagen proportions including total, aggregated and distributed collagen percentages; collagen string properties such as the thickness, length, and width; and ratios of different collagen string types. See Table 1 and Supplementary Table S1 for details.

**Table 1.** Characteristics evaluated in the study and their explanation.

Characteristics	Explanation
String	Known as collagen fiber, strip structure. These structures have specific attributes in themselves (including short, long, thin, thick string, string area, length, width, string eccentricity, solidity, perimeter, orientation), and quantitation attributes, which reflect morphological characteristics of collagen accurately, to perform quantitative morphological assessment of fibrosis dynamics.
Aggregated	Collagen was processed with fibrosis, some were aggregated and formed new structures (collagen fiber). Collagen fibers contained morphological characteristics, which were quantified, and the degree of fibrosis and fibrosis dynamics were then estimated.
Distributed	Collagen was processed with fibrosis, and some were scattered in tissue, forming tiny collagen fiber that contained morphological characteristics, which were quantified, and the degree of fibrosis and fibrosis dynamics were then estimated.
Portal	Consisted of portal tract (including the hepatic vein, one hepatic artery and one bile duct), central vein, and other lumens (lymph-vessel, nerve branch etc.). Pathological outer layers were adhered to a large number of collagen, according to the morphological characteristics of portal collagen fibers, which were quantified, and the degree of fibrosis and fibrosis dynamics were then estimated.
Septa	Complete septa linked some portal to portal tracts and bridged some portal tracts to central veins, forming a special morphological characteristic called “septa”, and collagen fibers with various features were quantified, and after, the degree of fibrosis and fibrosis dynamics were estimated.
Fibrillar	Tissue fibrosis, (except portal and septa fibrosis). Fibrillar fibrosis resulted in collagen fiber, which also had one important feature from hepatic fibrosis sinus cells, fibrosis of extracellular matrix. Morphological characteristics were quantified, and the degree of fibrosis and fibrosis dynamics were then estimated.
Cross-link	Collagen fibers that were X-bracing in some way in the process of fibrosis. Confirming the number of nodes is helpful for early liver fibrosis progression evaluation.

### Statistical analysis

The qFibrosis parameters for patients with CHB, PBC and NASH were analyzed. One-way ANOVA test was also used for parameter comparison between different fibrosis stages. In order to determine the characteristics of liver fibrosis from different etiologies, Spearman correlation analysis was used to analyze correlation between parameters and stages.

## Results

Parameters of aggregated collagen in portal, septal and fibrillar areas all increased significantly with higher fibrosis stages in samples from PBC and CHB (P<0.05), but parameters of distributed collagen did not increase significantly (P>0.05). There was no significant increase in parameters in samples from NASH (P>0.05) (Figure 1).

**Figure 1.** Results of one-way ANOVA analysis of parameters in portal, septal and fibrillar areas with liver fibrosis stages in samples from chronic hepatitis B (CHB), primary biliary cirrhosis (PBC), and non-alcoholic steatohepatitis (NASH). Orange, light blue and gray colors are used for differentiation of different parameters. SHG, second harmonic generation; AGG: aggregated collagen percentage; DIS: distributed collagen percentage. See Supplementary Table S1 for details.

Spearman correlation analysis showed a significant correlation between parameters in portal, septal and fibrillar areas for both CHB and PBC samples (P<0.05), but no significant correlation was found between collagen parameters and stage of liver fibrosis for both CHB and PBC samples (P>0.05). There was no significant correlation between NASH parameters and fibrosis stages (P>0.05) (Figure 2).

**Figure 2.** Spearman correlation analysis of parameters in portal, septal and fibrillar areas with stages for chronic hepatitis B (CHB), primary biliary cirrhosis (PBC) and non-alcoholic steatohepatitis (NASH). Orange, light blue and gray colors are used for differentiation of different parameters. SHG, second harmonic generation; AGG, aggregated collagen percentage; DIS, distributed collagen percentage. See Supplementary Table S1 for details.

For CHB and PBC patients, the highest correlation was between the septal parameters and stages of fibrosis, in the middle was the correlation between portal parameters and stages, and the lowest correlation was between fibrillar parameters and stages, which suggest that the septal parameter is the most important for predicting liver fibrosis progression (Figure 3).

**Figure 3.** Correlation of parameters and stages of liver fibrosis in samples from chronic hepatitis B (CHB) and primary biliary cirrhosis (PBC).

From the second harmonic generation and two-photon excited fluorescence images, the pathological patterns of fibrosis are different in different etiologies, with collagen stained in green and liver cell structure stained in red (Figure 4).

**Figure 4.** Second harmonic generation and two-photon excited fluorescence images of different patterns of fibrosis by different etiologies. Collagen is stained green and liver cell structure is stained red. *A*, Primary biliary fibrosis, in which fibrosis began in portal tracts (arrow). *B*, Chronic hepatitis B, in which expanded portal tracts are linked by fibrous tissue and slender bridge septa are connected to a portal tract and central vein (arrows). *C*, Non-alcoholic steatohepatitis, showing pericellular fibrosis, fibrous lattice surrounding individual and small groups of hepatocytes and vacuoles cells (arrows).

## Discussion

Liver biopsy is still the gold standard in etiology differentiation and severity evaluation of liver fibrosis, providing descriptive diagnosis. By analyzing pathological changes of liver diseases, researchers establish disease severity according to pathological characteristics, such as necrosis in portal or septal area, degeneration or foci necrosis in fibrillar area, portal veins inflammation and liver fibrosis (13). In order to differentiate mild from severe liver diseases with a semi-quantitative analysis, pathological changes such as liver tissue inflammation and fibrosis have been given scores. However, it is reported that the intra- and inter-observer discrepancy in the available semi-quantitative systems can be as high as 35% (15 [Bibr B16]–17).

Effort is made to assess the progression of liver fibrosis by the proportion of collagen fibers in the liver. Morphological assay (morphometry) is frequently used in clinical studies. In this method, collagen fibers from a stained area are calculated and compared with the whole area under analysis to get the collagen proportionate area (CPA). CPA, also called collagen area ratio, is 1 to 7% in normal liver and 12 to 36% in liver cirrhosis. CPA can be further subdivided, and it is used as an independent predictor for cirrhosis (18). Despite of this, CPA is still inconsistent and subjective to some extent, and showed drastic changes only in advanced stages of fibrosis, and was unable to differentiate between early stages (6).

qFibrosis quantitative analysis of liver biopsies includes quantitative and structural information of fibrosis, which can reflect changes of fibrosis intensity and distribution. Combining the staging method with fully quantitative fibrosis analysis can also solve the problems of the traditional stage system - etiology differentiation and fibrosis reversion. The fully quantitative method can confirm fibrosis reversion from a pathological point of view.

In this study, we assessed the performance of qFibrosis for the evaluation of fibrosis and histological stages in chronic cholestatic diseases of PBC, CHB, and NASH. We found that the parameters of aggregated collagen in portal, septal and fibrillar areas all increased significantly with higher stages of liver fibrosis in PBC and CHB, but the parameters of distributed collagen did not significantly increase in the same samples. Also, there was a significant correlation between parameters in portal, septal and fibrillar areas for both CHB and PBC, but not between the collagen parameters and the stages of liver fibrosis in those diseases. There was no significant correlation between NASH parameters and fibrosis stages. For CHB and PBC patients, the highest correlation was between septal parameters and fibrosis stages, the second highest was between portal parameters and fibrosis stages and the lowest correlation was between fibrillar parameters and fibrosis stages, which suggest that the septal parameter was the most important predictor for liver fibrosis progression.

Compared with parameters of distributed collagen, parameters of aggregated collagen in portal, septal and fibrillar areas seem to be more suitable for assessment of liver fibrosis progression in PBC and CHB patients. Pathologically, for PBC patients, liver fibrosis progression happens in the septal area, although it starts in the portal area. For CHB, parameters in the portal and septal areas were strongly correlated with progression of stages, which suggests that the parameters in these two areas, particularly the aggregated collagen parameters, could be used in the assessment of liver fibrosis progression and reversion. The qFibrosis candidate parameters based on CHB are also applicable for quantitative analysis of liver fibrosis in PBC. In this study, the parameters for NASH were not significantly correlated with fibrosis stages, suggesting that the candidate parameters of qFibrosis based on CHB are not suitable for quantitative assessment of liver fibrosis in NASH. Further studies are necessary to reach a stronger conclusion, because of the small sample size of NASH cases in this study.

## Supplementary Material

Click here to view [pdf]
